# The Effect of an Educational Intervention on Oral Health Literacy, Knowledge, and Behavior in Iranian Adolescents: A Theory-Based Randomized Controlled Trial

**DOI:** 10.1155/2022/5421799

**Published:** 2022-06-06

**Authors:** Fatemeh Movaseghi Ardekani, Faezeh Ghaderi, Mohammad Hossein Kaveh, Mahin Nazari, Zakieh Khoramaki

**Affiliations:** ^1^Department of Health Promotion, Faculty of Health, Shiraz University of Medical Sciences, Shiraz, Iran; ^2^Department of Pediatric Dentistry, Faculty of Dentistry, Shiraz University of Medical Sciences, Shiraz, Iran; ^3^Research Center for Health Sciences, Institute of Health, Department of Health Promotion, School of Health, Shiraz University of Medical Sciences, Shiraz, Iran; ^4^Student Research Committee, Department of Health Promotion, School of Health, Shiraz University of Medical Sciences, Shiraz, Iran

## Abstract

**Introduction:**

Oral health is one of the most important issues in public health. Most educational interventions, as the primary prevention strategy, are focused on increasing information and knowledge and are not usually effective. Therefore, the present study is aimed at determining the effect of theory-based education on oral health behavior and its psychological determinants including dental health literacy.

**Method:**

This randomized controlled educational trial was conducted in two girls' high schools that were selected by multistage cluster sampling and were divided into an intervention and a control group. Literacy, knowledge, oral health behavior, dental plaque index, and constructs of the protection motivation theory were evaluated before and one month after four training sessions. Finally, the data were entered into the SPSS 19 software and were analyzed using the chi-square test, independent *t*-test, and Mann–Whitney test at the significant level of 0.05.

**Result:**

Before the intervention, there was no significant difference between the intervention and control groups regarding the mean scores of knowledge, behavior, and oral health literacy; plaque index; and protection motivation theory constructs. After the educational intervention, however, the means of these variables were significantly improved in the intervention group compared to the controls (*p* < 0.05).

**Conclusion:**

The study findings were in favor of the effectiveness of the theory-based educational intervention in improving the knowledge, literacy, and behavior related to oral health. Yet, further research is suggested to determine the effectiveness of such an intervention in male students as well as in populations with different socioeconomic and cultural statuses.

## 1. Introduction

Oral health is central to a person's overall health and well-being [1]. Poor oral health directly affects many aspects of life including functional, aesthetic, nutritional, and psychological problems [2]. Oral diseases are also accompanied by serious health and economic burdens and impose large economic burdens on families and healthcare systems [3]. These diseases can disturb individuals' well-being and self-esteem, as well [4]. Despite its preventable nature, it is still one of the costliest diet- and lifestyle-related diseases. The cost of treating dental decay alone can easily exhaust a country's total healthcare budget for children [5]. In spite of a general reduction in dental caries in all ages, studies have shown that it has remained high during adolescence. According to the World Health Organization's (WHO) report, approximately 60–90% of school-age children suffer from dental caries. In the Mediterranean region, the Eastern Mediterranean region including Iran has shown the highest mean for decayed, missing, and filled teeth (DMFT) [6, 7]. Disparities in oral health status can be determined by such factors as the socioeconomic, cultural, and educational status; access to and use of healthcare services; oral health literacy; and the related behaviors [8].

Evidence has revealed a significant relationship between the oral health status and oral health literacy. In other words, promotion of oral health literacy can help reduce the difference among various groups regarding the oral health status [9, 10]. Studies have also indicated a relationship between low levels of oral health literacy and a higher prevalence of dental caries, tooth loss, and periodontal disease [11]. Oral health literacy is a more specific aspect of the broad concept of health literacy. Health literacy is related to individuals' literacy, knowledge, motivation, and skills to access, understand, evaluate, and use health information in order to make decisions about obtaining health care and promoting health [12]. Oral health literacy is the degree to which individuals have the capacity to obtain and process basic oral health information and services needed to make appropriate health decisions [13]. In fact, oral health literacy is a fundamental commitment to assisting patients become full participants in their own health care [14]. It can also lead to oral health by facilitating access to oral health information, the ability to evaluate the existing information, the effective use of information, and informed decision making [15]. Therefore, low levels of health literacy may be associated with fewer preventive services, delays in diagnosing medical conditions, poor adherence to medical guidelines, poor self-management skills, and higher medical costs [16]. Studies also demonstrated that adequate oral health literacy was strongly associated with a better oral health status in all groups [17, 18].

Among age groups, adolescence is a crucial stage in human development and oral health plays an important role in this period. The risk for caries, traumatisms, and periodontal diseases increases in adolescents compared to younger children due to the tendency to poor eating habits. Therefore, it is necessary to develop specific preventive strategies for this population [19].

Studies conducted on oral health literacy in Iran and the world have shown that more than half of adults do not have sufficient oral health literacy. Thus, the WHO has considered the improvement of oral health literacy through planned educational interventions as a priority [8, 20, 21]. Effective education is an essential component and an important prerequisite for achieving the goals of oral health promotion programs [22–24]. Evidence has proved the higher effectiveness of traditional education methods compared to model-based ones, because model-based education involves the factors that are more effective in behavior change [25, 26]. In other words, theory-based educational intervention can lead to effective training through understanding the causes of the problem, providing an approach to achieving the goal, and identifying what is to be achieved at the end of the program [24].

One of the prominent theories of behavior change is the protection motivation theory (PMT). According to this theory, individuals' understanding is the best predictor of behavioral intention and “threat appraisal” and “coping appraisal” are necessary to motivate people to engage in health-related behaviors [27]. In PMT, the threat appraisal components include (1) perceived severity (a person's estimation of the severity of a disease) and (2) perceived vulnerability (a person's estimation of the probability of the disease incidence). Additionally, the components of coping appraisal include (1) response efficacy (an individual's expectancy that implementing the recommendations can remove a threat), (2) self-efficacy (belief in one's ability to carry out a recommended plan of action successfully), and (3) response cost (beliefs about how costly performing the recommended response will be to the individual). This theory has been used for analyzing or designing educational interventions for behaviors such as oral health [28] and physical activity [29] and determining the predictive factors for preventing smoking [30], preventing malaria [26], and preventing agricultural injuries in children [31, 32] (Figure 1).

As mentioned earlier, oral health behaviors play a key role in the general health of individuals, especially children and adolescents, and it is vitally important to start healthy habits at early ages. Additionally, numerous studies have reported a relationship between oral health literacy and oral health status. Hence, the present study is aimed at investigating the role of education using the PMT in improving oral health literacy and oral health behaviors in high school students in Shiraz.

## 2. Materials and Methods

This randomized controlled trial was performed using a theory-based educational intervention in 2017 in order to investigate the role of education based on the PMT in improving oral health literacy and oral health behaviors among high school girls (14–15 years old) in Shiraz, Fars province, Iran.

Using the following formula, based on a similar previous study [33] and considering (*μ*_1_ − *μ*_2_) = 7.67, *σ* = 6.56, first type error of 5%, and test power of 80%, 90 people were estimated for each study group. Considering a loss rate of 20%, the sample size was increased to 180 individuals (90 in the intervention group and 90 in the control group). The participants were selected via multistage cluster sampling. During the study, 18 individuals (13 in the intervention group and 5 in the control group) were excluded due to failure in cooperation. Finally, 162 students were divided into the intervention (*n* = 77) and the control (*n* = 85) groups.

(1) $$\begin{array}{c} n=\frac{{\left(Z_{1-a/2}+Z_{1-\beta }\right)}^{2}\left(S_{1}^{2}+S_{2}^{2}\right)}{{\left(\mu_{1}-\mu_{2}\right)}^{2}}. \end{array}$$

In the first phase, the four educational districts in Shiraz were randomly classified into two categories (1 and 2 in one category and 3 and 4 in the other category). Then, from each district, one district was selected randomly (2 and 4(. Afterwards, two schools were selected from each district (four schools in total) and were randomly divided into the intervention and control groups. Finally, one class was randomly selected from each school and enrolled into the study (four classes in total). In order to prevent information leakage between the intervention and control groups, random allocation was done at the cluster (i.e., school) level.

The inclusion criteria of the study were being a ninth-grade female student (aged 14–15 years), studying in governmental schools, and being willing to cooperate. Written informed consent forms were also obtained from the participants and their parents before the trial.

### 2.1. Research Tools

The data were collected using two researcher-made questionnaires based on the PMT constructs and oral health literacy. One questionnaire was used to assess the participants' demographic information, knowledge, oral health behaviors, and the PMT constructs, while the second one was utilized to evaluate their oral health literacy. The participants were required to fill out the questionnaires before and one month after the training intervention.

The questionnaires were designed using valid scientific sources [8, 24, 34, 35]. The first part of the first questionnaire included demographic information (student's age and parents' levels of education and occupations). The second part was related to the assessment of knowledge using 11 questions, assigning one score to “correct” answers and zero scores to “incorrect” or “I do not know” answers. In the third section, the participants' oral health behaviors were assessed through nine self-report questions including brushing activities (such as frequency, duration, time, and aids), having checkups by a dentist (such as regularity and reason), and type of food intake. In the next part, 50 items with a five-point Likert scale (ranging from “strongly disagree” to “strongly agree”) were used to evaluate the PMT constructs.

In the second questionnaire, 25 items with a five-point Likert scale were used to measure eight dimensions of oral health literacy, i.e., reading, understanding, apprising, communicating, applying, accessing, listening, and numeracy skills. It is worth mentioning that four questions were extracted from the questionnaire designed by Naghibi et al. with the permission of the authors [34].

The Cronbach's alpha coefficient was calculated as 0.74 for the first questionnaire and 0.83 for the oral health literacy questionnaire. Their validity was also approved by experts and faculty members at faculties of health and dentistry (CVI = 0.96, CVR = 0.99) (Table 1).

The questionnaires were completed by the participants before and one month after the intervention. In addition, the dental plaque index was evaluated by the researcher at both times.

The intervention group received four one-hour educational intervention sessions on knowledge, behavior, and oral health literacy based on the PMT framework. These sessions were held once weekly for four weeks. However, the control group did not receive any training programs.

Before designing the educational intervention, the contents of the school textbooks were reviewed. The oral health content was found to be very limited, focusing on factual information rather than addressing behavioral determinants and skills. Besides, there was no content on oral health literacy in the textbooks. The educational content was designed based on the results of the pretest as well as a review of the related scientific texts [36–38]. It addressed such topics as oral structure; common terms in dentistry; role of microbial plaques; methods of brushing and flossing; importance of regular referrals to dentists; healthy diet; appropriate use of fluoride; essential tips for choosing a toothbrush, toothpaste, and other oral hygiene items; and reliable sources of information in the field of oral health. Due to the students' engagement in the learning process, in addition to using the lecture method, usage was made of active learning techniques such as group discussion, group work, role playing, and puzzle. Educational technologies such as video clips, photos, educational booklets, and posters were used, as well. On the first day of the intervention, toothbrushes and fluoride-containing toothpastes were distributed among all the participants. At the end of the research project, the educational booklet was given to the control group participants (Table 2).

The data were entered into the SPSS 19 software and were analyzed using descriptive statistics, independent sample *t*-test, paired sample *t*-test, Mann–Whitney *U* test, Wilcoxon signed-rank test, Pearson's correlation, and linear regression analysis. The significance level was set at *p* < 0.05.

## 3. Results

This study was initiated with 180 adolescents enrolled from four randomly selected schools in the study area. Data from 18 students were excluded from the study due to incomplete questionnaires, refusal to continue cooperation, and absence from the educational program. Thus, the data of 162 students who participated in the educational program were analyzed. The mean (SD) age of the participants was 14.71 ± 0.45 years in the intervention group and 14.66 ± 0.47 years in the control group.

Before the intervention, the results of the chi-square test revealed no significant difference between the control and intervention groups regarding age, household size, and mother's occupation (*p* < 0.05). Although random distribution was used for sampling, there was a significant difference between the two groups with regard to father's occupation and parents' education levels (Table 3). The Pearson's correlation test did not show any significant relationships between oral health knowledge and behavior and household size, parents' education levels, and parents' occupations. The results also revealed no significant relationships between oral health literacy and household size, parents' education levels, and mother's occupation. Among the demographic variables, there was a significant negative correlation between oral health literacy and father's occupation (Table 4).

The results indicated a significant positive correlation between the father's education level and the student's appraising skills; the mother's education level and the student's perception and assessment; and the mother's occupation and the student's appraising skills. There was also a significant negative relationship between the father's occupation and the student's perceptual skills.

Among the oral health literacy components, the highest mean score was related to reading skills (85.4%) in the intervention group and communication skills (83.5%) in the control group. On the other hand, the lowest mean score was related to appraising skills in both groups (65.2% in the intervention group vs. 62% in the control group). In order to investigate the relationship between oral health literacy skills and oral health-related behaviors, Pearson's correlation coefficient was used. The results revealed the highest correlation between oral health-related behaviors and applying, appraising, numeracy, and listening skills.

Before the intervention, there was no significant difference between the intervention and control groups regarding the mean scores of oral health knowledge, oral health behaviors, and oral health literacy. After the intervention, however, the difference between the two groups was statistically significant (Table 5).

The results of the paired sample *t*-test showed no significant difference between the two groups regarding the mean score of the dental plaque index before the intervention. After the intervention, however, a significant difference was observed between the two groups in this regard. Although the mean scores of the dental plaque index decreased in both groups after the intervention, the decrease was more prominent in the intervention group (Table 5).

In this study, the two groups were compared in terms of changes in the mean scores of the PMT constructs (perceived vulnerability, perceived severity, response costs, response efficacy, self-efficacy, and cues to action) before and one month after the intervention. The results showed no significant difference between the two groups regarding the mean scores of the constructs before the intervention. Nonetheless, a significant difference was observed between the two groups in this respect after the intervention. Moreover, the mean scores of the constructs were significant before and after the educational intervention in the intervention group, but not in the control group (Table 5).

## 4. Discussion and Conclusion

The present randomized controlled trial was designed not only to assess the effect of a theory-based educational intervention on improving knowledge and oral health literacy but also to improve the oral health-related behaviors through promoting knowledge and health literacy. The results revealed no significant relationship between the demographic variables and oral health knowledge and behaviors. Up to now, most studies have explored the role of demographic factors in oral health status rather than knowledge or behavior. El-Qaderi and Taani [39] reported that the mother's education level was not significantly related to the student's knowledge. Similarly, Qiu et al. [40] found no associations between the caregiver's social support and the child's oral health-related behaviors. In contrast, Wierzbicka et al. [41] came to the conclusion that children's dental care habits (behaviors) were highly influenced by the mothers' education levels. This contradiction might be due to the differences in the participants' age and the utilized tools. In Poutanen et al.'s research [42], the parents of the children whose oral health behaviors were favorable were more likely to have a high-level occupation. Kassak et al. [43] also demonstrated that the father's education level was significantly correlated to the frequency of tooth brushing among the students. Nonetheless, Apolinario et al. [44] conducted a study entitled “detecting limited health literacy in Brazil” and showed that the father's occupation and level of education were not the predictors of health literacy. Hirvonen et al. [45] also carried out a research entitled “sociodemographic characteristics associated with the everyday health information literacy of young men” and found that the father's manual labor and mother's professional occupation decreased the odds of having high health information literacy. The discrepancy among the results might be explained by different demographic classifications as well as the investigation of demographic variables alongside some behaviors and oral health knowledge.

In this study, among the components of oral health literacy, the highest mean score was related to reading skills in the intervention group and communication skills in the control group. On the other hand, the lowest mean score was related to assessment skills in both study groups. Although no similar study was found to compare the dimensions of oral health in adolescents, a study performed by Naghibi et al. [8] in adults showed that most participants had high arithmetic skills but poor reading skills. Most studies have also shown low health literacy and oral health literacy in the community [8, 20, 46–48]. In another research conducted by Kaboudi et al. [49], the participants scored high in comprehension skills, but low in reading skills. In Haerian et al.'s study also [15], among the dimensions of oral health literacy, reading was more prominent. The observed discrepancy may be attributed to different age groups as well as the utilized tools. The abovementioned studies were conducted on adults, while Haerian et al.'s research and the present one were performed on a limited age group.

The present study results revealed a decrease in the mean plaque index in both study groups after the educational intervention, but this decrease was more prominent in the intervention group. Consistently, the review studies performed by Hajimiri et al. [50], SohrabiVafa et al. [51], and Decrose [23] indicated a decrease in the dental plaque index in both groups after the intervention. Nevertheless, the decrease was more prominent in the intervention group, which confirmed the role of education. The reduction in the dental plaque index in this study might be due to the motivational role of the questionnaire in the control group, which may not continue in the long run.

The current study compared the two groups regarding the mean changes in the scores of the PMT constructs in the field of oral health behaviors before and after the intervention. The results showed a significant change in the intervention group's mean scores before and after the educational intervention. Review of the literature revealed only one study on the impact of PMT on the promotion of oral health-related behaviors. That study was done by Kimhasawad et al. on 102 children aged 9–18 months and their caregivers based on an oral health education program in 2021. The results indicated that the caregivers' perceptions of the severity of premature carious lesions in children and their belief in self-efficacy were significantly higher in the intervention group than in the control group in a 12-month follow-up [28]. The present study also revealed similar results among the adolescents in the intervention group. Due to the similarity of some PMT constructs to those of the health belief model, the studies performed using this model were used for comparison. Hajimiri et al. [50] reported a significant change in the constructs of the health belief model after the educational intervention, while no significant changes were detected in the control group. These results were in line with those of the present investigation. In the study conducted by Kakudate et al. [52], compared to traditional training, training based on a six-step behavioral cognitive method led to the improvement of self-efficacy in the intervention group, while no significant changes were observed in the control group. Overall, the changes in the PMT constructs might result from the educational intervention carried out on the basis of this model.

To the best of our knowledge, this was the first theoretical empirical study on oral health behaviors and its determinants including dental health literacy amongst high school girls. Another strength of the study was the evaluation of the dental plaque index, as an objective criterion for compensating the possible bias associated with the students' responses. However, this study had several limitations. Firstly, this study was performed on female students and the results may not be generalizable to male students. It should be noted that Iran's education policy has considered restrictions on the presence of researchers or teachers of the opposite sex at schools. Besides, enrollment of male students into the study required a larger sample size and a larger number of schools, which were not possible considering the time and resources allocated to this MSc thesis. Another limitation of the study was the employment of self-report measures, which might be accompanied by some social desirability biases. Therefore, the dental plaque index was evaluated as an objective criterion for compensating for the possible self-report bias.

In conclusion, oral health literacy is a new issue that is necessary for the promotion of oral health. Theory-based educational interventions can increase self-care and self-efficacy and be effective in promoting knowledge, literacy, and oral health-related behaviors. Yet, future long-term studies are recommended to assess behaviors and oral health. Further studies are also suggested to determine the effectiveness of such interventions in different groups of students in terms of age, gender, and socioeconomic and cultural statuses.

## Figures and Tables

**Figure 1:** Protection motivation theory (modified from [32]).

**Table 1:** Questionnaires based on the protection motivation theory constructs and oral health literacy.

PMT constructs	Example of items	Options	Number of items	Range of scores	Cronbach's alpha
Perceived vulnerability	I look ugly with yellow and rotten teeth.	1 = strongly disagree, 2 = disagree, 3 = no idea, 4 = agree, 5 = strongly agree	8	8–40	0.65
Perceived severity	If I do not brush my teeth, I may have decayed teeth and gum disease.		9	9–45	0.70
Response costs	I do not go because of the high cost of dentistry.		10	10–50	0.74
Response efficacy	If I spend enough time on my oral health, I will look more beautiful.		6	6–30	0.72
Self-efficacy	I floss even when I am at a party or traveling.		11	11–55	0.87
Cue to action	Seeing general education materials in public places encourages my oral hygiene.		6	6–30	0.67

**Table 2:** Organization of the educational sessions in the intervention group.

Meeting	Contents	Methods (learning activities)	Educational technology tools	Measuring tools )evaluation strategy)
First	Definition of oral health and oral health literacy; providing statistics on the prevalence of oral diseases in Iran and the world; the effect of oral diseases on reducing a person's quality of life; familiarity with oral structure and common terms in dentistry (emphasis on perceived severity, perceived vulnerability, reading, and understanding dimensions)	Teaching-learning, interactive lectures, and question and answer	Magic boards, photos, video projectors (PowerPoint), dental modeling	Preparing a report on the oral condition of family members
Second	Explaining oral diseases and their causes; the relationship between oral health literacy and oral health status (emphasis on perceived severity, response efficacy, reading, and perceptual dimensions)	Teaching-learning, group discussion	White boards, markers, photos, video projectors (PowerPoint)	Preparation of a list of barriers
Third	Explaining strategies for oral health literacy promotion and disease prevention and control, identifying barriers, and finding ways to overcome them (emphasis on response efficiency, response cost, applying, and oral health literacy performance)	Group discussion, brainstorming	Video projector (PowerPoint), photos, preventive devices (toothbrush, floss, mouthwash), poster, puzzle	Making a list of solutions to overcome barriers in the classroom and preparing posters
Fourth	Introduction oral hygiene devices and sources for obtaining oral health information (emphasis on self-efficacy, communication, evaluation, computational dimension (numeracy and listening skills), and familiarity with reliable sources of health literacy	Demonstration method, lecture	White board and marker, video projector (PowerPoint), tooth modeling, and preventive devices (toothbrush, floss, mouthwash)	Preparing a list of sources for obtaining information on oral health literacy

**Table 3:** Demographic characteristics of the participants in the intervention (*n* = 77) and control (*n* = 85) groups at baseline.

Variables	Category	*n* (%) intervention	*n* (%) control	*p* value^∗^
Age (years)	14	26 (33.76)	24 (23.28)	0.447
	15	51 (66.24)	61 (71.76)	
Household size	3	5 (6.5)	12 (14.1)	0.187
	4	43 (55.8)	36 (42.4)	
	5	25 (32.5)	26 (30.6)	
	≥6	4 (5.2)	11 (13)	
Father's level of education	Low (up to secondary school)	8 (10.4)	38 (44.7)	0.000
	High school and diploma	40 (52)	30 (35.3)	
	Academic	29 (37.7)	17 (20)	
Mother's level of education	Low (up to secondary school)	15 (19.5)	37 (43.6)	0.003
	High school and diploma	39 (50.7)	35 (41.2)	
	Academic	23 (29.9)	13 (15.6)	
Father's occupation	Unemployed/worker/retired or dead	15 (19.5)	19 (22.3)	0.047
	Self-employed	40 (52)	55 (64.7)	
	Governmental employee/doctor/engineer	22 (27.3)	11 (16.5)	
Mother's occupation	Homemaker/retired	59 (76.6)	74 (87)	0.087
	Worker/self-employed	7 (9.1)	5 (5.9)	
	Governmental employee/doctor/engineer	11 (14.3)	6 (7.1)	

^∗^Chi-square.

**Table 4:** The results of Pearson's correlation test among the demographic characteristics.

		Age (years)	Household size	Father's level of education	Mother's level of education	Father's occupation	Mother's occupation	Oral health knowledge	Oral health behavior	Oral health literacy
Age (years)	Pearson correlation	1								
	Sig. (2-tailed)									
Household size	Pearson correlation	0.011	1							
	Sig. (2-tailed)	0.889								
Father's level of education	Pearson correlation	−0.181^∗^	−0.153^∗^	1						
	Sig. (2-tailed)	0.018	0.047							
Mother's level of education	Pearson correlation	−0.043	−0.226^∗∗^	0.710^∗∗^	1					
	Sig. (2-tailed)	0.576	0.003	0.000						
Father's occupation	Pearson correlation	−0.041	−0.118	0.174^∗^	0.097	1				
	Sig. (2-tailed)	0.594	0.127	0.023	0.208					
Mother's occupation	Pearson correlation	0.002	−0.147	0.294^∗∗^	0.448^∗∗^	−0.087	1			
	Sig. (2-tailed)	0.984	0.056	0.000	0.000	0.260				
Oral health knowledge	Pearson correlation	−0.104	0.035	0.019	0.092	−0.033	.038	1		
	Sig. (2-tailed)	0.178	0.647	0.802	0.235	0.666	.625			
Oral health behavior	Pearson correlation	−0.050	−0.065	0.130	0.104	−0.118	.085	.256∗∗	1	
	Sig. (2-tailed)	0.517	0.398	0.091	0.176	0.127	.271	.001		
Oral health literacy	Pearson correlation	−0.060	0.027	0.124	0.135	−0.154^∗^	.125	.265∗∗	.355∗∗	1
	Sig. (2-tailed)	0.441	0.727	0.109	0.080	0.046	.105	.000	.000	

^∗^Correlation is significant at the 0.05 level (2-tailed). ^∗∗^Correlation is significant at the 0.01 level (2-tailed).

**Table 5:** Comparison of the means of changes in the variables in the two groups before and one month after the intervention.

Variable	Group	Preintervention	Postintervention	Difference mean ± SD	Sig.
		Mean ± SD	Mean ± SD		
Knowledge	Control	4.87 ± 1.91	5.98 ± 2.03	1.11 ± 1.90	<0.05^∗^
	Intervention	5.25 ± 2.08	11.83 ± 1.18	6.57 ± 2.15	<0.05^∗^
	Sig.^a^	0.37	<0.001^∗∗∗^	<0.05^∗^	
Behavior	Control	14.74 ± 3.24	15.03 ± 2.89	0.29 ± 1.80	0.137
	Intervention	15.45 ± 3.87	17.51 ± 3.59	2.06 ± 2.56	<0.000^∗∗∗^
	Sig.^b^	0.205	<0.001^∗∗∗^	<0.05^∗^	
Oral health literacy	Control	80.57 ± 10.02	81.92 ± 9.11	6.76 ± 1.35	0.069
	Intervention	82.64 ± 11.58	94.83 ± 10.61	10.02 ± 12.18	<0.000^∗∗∗^
	Sig.^a^	0.224	<0.001^∗∗∗^	<0.05^∗^	
Dental plaque index	Control	2.20 ± 0.66	1.98 ± 0.69	−0.21 ± 0.48	0.035^∗^
	Intervention	2.02 ± 0.59	0.83 ± 0.75	−1.96 ± 0.58	0.000^∗∗∗^
	Sig.^b^	0.080	<0.001^∗∗∗^	<0.05^∗^	
Perceived vulnerability	Control	22.94 ± 4.20	23.49 ± 4.31	0.55 ± 4.25	0.400
	Intervention	23.44 ± 3.16	27.75 ± 4.20	4.31 ± 0.33	0.000^∗∗∗^
	Sig.^b^	0.391	<0.001^∗∗∗^	<0.05^∗^	
Perceived severity	Control	26.29 ± 5.28	26.56 ± 4.91	0.27 ± −4.76	0.365
	Intervention	27.19 ± 4.55	30.71 ± 3.84	3.51 ± 3.74	<0.000^∗∗∗^
	Sig.^b^	0.250	<0.001^∗∗∗^	<0.05^∗^	
Response costs	Control	15.11 ± 6.97	15.70 ± 7.04	0.58 ± 3.96	0.291
	Intervention	15.80 ± 6.52	13.10 ± 6.06	−2.70 ± 5.54	0.008^∗∗^
	Sig.^b^	0.519	<0.013	<0.05^∗^	
Response efficacy	Control	21.23 ± 2.50	21.35 ± 2.35	0.11 ± 2.50	0.373
	Intervention	20.84 ± 2.89	22.50 ± 2.11	1.66 ± 3.03	<0.000^∗∗∗^
	Sig.^a^	0.498	<0.001^∗∗∗^	<0.05^∗^	
Self-efficacy	Control	22.88 ± 9.66	26.32 ± 8.50	3.44 ± 6.87	0.992
	Intervention	23.50 ± 8.59	30.87 ± 7.25	7.36 ± 7.42	<0.000^∗∗∗^
	Sig.^b^	0.666	<0.001^∗∗∗^	<0.05^∗^	
Cues to action	Control	16.16 ± 3.79	16.84 ± 4.32	0.68 ± 3.44	0.138
	Intervention	15.54 ± 4.57	20.42 ± 3.31	4.88 ± 4.11	<0.000^∗∗∗^
	Sig.^b^	0.349	<0.001^∗∗∗^	<0.05^∗^	

^∗^ *P* < 0.05, ^∗∗^*P* < 0.01, ^∗∗∗^*P* < 0.001; ^a^Mann–Whitney *U* test; ^b^*t*-test.

## Data Availability

The data used to support the findings of this study are included within the article.
